This article has been retracted.

# A Study on the Evaluation of Polyenoic Vegetable Oils and Their Female Health Benefits Based on Time Series Analysis Model: The Case of Peony Seed Oil

**DOI:** 10.1155/2022/3127698

**Published:** 2022-03-25

**Authors:** Haibo Li, Songhao Kang, Lijuan Sun

**Affiliations:** ^1^Shengnong Technology Group, Jinzhong, Shanxi 030805, China; ^2^College of Engineering, China Agricultural University, Haidian, Beijing 100083, China; ^3^Beijing Madixin Food Technology Co,Ltd., Haidian, Beijing 100036, China

## Abstract

Polyenoic vegetable oils mainly contain polyenoic acids such as linoleic acid and linolenic acid, as well as active ingredients such as VE, phytosterols, mineral elements, and squalene. Among them, schisandra oil, kiwi seed oil, grape seed oil, maitake fruit oil, and evening primrose seed oil all contain up to 80% or more polyenoic acids. Studies have shown that polygenic vegetable oils have the effects of assisting in lowering blood lipids, antioxidation, delaying ageing, anti-inflammation, sun protection, moisturizing, slimming and weight loss, etc. They can be widely used in nutritional and healthy edible oils, health food, skin care, and cosmetic products and have great prospects for development and utilization. This paper explores the application of artificial neural networks in the analysis of data. A nonlinear time series prediction method based on the BP algorithm is proposed. The prediction accuracy is much higher than that of the traditional method.

## 1. Introduction

A valuable medicinal and food plant, rich in protein, traces elements and vitamins; peony flowers have been used since the Song Dynasty to make pastries, tea, and various dishes [1]. In addition, peony flowers have been used to treat menstrual disorders and dysmenorrhea in women. With the development of the time, peonies have not faded out of sight, but are increasingly valued by people. In 2013, Heze “Feng Dan” was approved by the State Ministry of Health as a new food ingredient. M. Peony flower essential oil is taken from peony petals and is a clear, transparent, aromatic, and volatile liquid. Because of its high cost, peony flower essential oil is also known as “liquid gold.” Peony flower essential oil is rich in aroma, natural, and safe, with a variety of antioxidant components, and is an emerging indigenous plant essential oil [2]. Peony flower essential oil is still in its infancy in China, and research on peony flower essential oil is still scarce, mainly focusing on the extraction method, composition, and antioxidant properties of peony flower essential oil [3].

Polygenic vegetable oils are natural vegetable oils extracted from the fruit, seed, and germ of plants that are mainly composed of polyunsaturated fatty acids (PUFA) and are also rich in VE, phytosterols, trace elements, and many other active substances [4]. In addition to the oleic and palmitic acids contained in common vegetable oils, polyunsaturated vegetable oils mainly contain polyunsaturated fatty acids such as linoleum and linoleum acids with two or more double bonds, such as grape seed oil, perilla oil, flaxseed oil, and kiwi seed oil [5, 6]. Therefore, polygenic vegetable oils can be used as edible oils to meet the intake requirements of human fatty acids, as well as for the production of pharmaceuticals and health foods, and as oily raw materials for cosmetics, with broad prospects for development and utilization [7].

At present, research on the efficacy of peony flower essential oil at home and abroad is still in its infancy, with studies mainly focusing on the antioxidant properties of peony flower essential oil and less on the other effects of peony flower essential oil [8]. The authors studied the antioxidant capacity of 14 different varieties of peony flower essential oils and found that all peony flower essential oils have certain antioxidant capacity, and among the 14 varieties, yellow peony and purple peony have the strongest antioxidant capacity, which is due to the fact that yellow peony and purple peony flower essential oils contain more terpenoids. In addition, peony flower essential oil also contains potent components such as phytol, oxygenated linalool, and farnesol, and it is speculated that peony flower essential oil may also have anti-inflammatory and antiplatelet activity and anticancer potential [9].

## 2. Related Work

As virgin crude oil of peony seed oil does not meet our standards for massage base oil, the crude oil of peony seed oil has to be refined. The common refining steps are generally filtration, degumming, deacidification, decolonisation, and depolarisation [10]. Filtration is mainly used to remove solid impurities from the gross oil by means of media with capillary pores or centrifugation. Degumming is used to remove colloidal impurities such as proteins, phospholipids, and mucilage from the oil. The presence of colloidal impurities can reduce the stability of the oil and can cause souring of the soil [11]. At present, commonly used degumming methods are intermittent hydration degumming and continuous hydration degumming. Deacidification, also known as alkali refining, is the process of adding calcium hydroxide, sodium hydroxide, or soda ash to make the free fatty acids in the oil react with the alkali to form soap horns and then removing the insoluble soap horns by filtration and centrifugation [12]. The common adsorbent materials used are activated carbon and activated white clay. After filtering, degumming, deacidification, and decolonisation of fats and oils, there are also special odours, which can be divided into three types: the odour of the different fats and oils themselves, the odour of the manufacturing and processing process, and the odour of the oxidation and decay of the fats and oils. The odour is discharged with water vapour. The decolonisation process is usually carried out under vacuum in order to reduce oxidation of the oil [13].

The content of unsaturated fatty acids in peony seed oil ranges from 82.00 to 93.00%, with linoleum acid, linoleum acid, and oleic acid being the most common of the unsaturated fatty acids [14]. We compared the fatty acid composition of peony seed oil with that of eight other common vegetable oils and found that the content of linoleum acid in peony seed oil was only slightly lower than that of linseed oil, but the total content of linoleum and linoleum acids was the highest among the nine vegetable oils. In addition to fatty acids, peony seed oil is also rich in phytosterols, squalene and vitamin E, and other unsaponifiables. The content of vitamin E in peony seed oil was also relatively high, reaching 9851 mg/100 g, which was higher than that of sesame oil (200–30.00 mg/100 g), olive oil (5.00–30.00 mg/100 g), camellia oil (24.90 mg/100 g), and wheat germ oil (103.40 mg/100 g) [15].

As an emerging woody plant oil, peony seed oil has no acute toxicity and geneticists and has high nutritional value and health effects. Peony seed oil is also rich in linoleum acid and linoleum acid, among which linoleum acid has the functions of cholesterol-lowering, blood lipid-lowering, immunity enhancement, antiallergy, antiaging, fat metabolism promotion, and liver cell regeneration [16]; linoleic acid has the functions of inhibiting cholesterol synthesis, anticancer, antioxidation, and prevention of diabetes. In addition, there are high levels of unsaponifiables in peony seed oil. Among the unsaponifiables, squalene and vitamin E, as natural antioxidants, have the functions of enhancing human immunity and antiaging; phytosterols are important intermediates of sterols and have the functions of lowering cholesterol and preventing atherosclerosis. The mineral elements present in peony seed oil also have important physiological functions and health effects, including maintaining the osmotic pressure of cell membranes, protecting the nerves, lowering cholesterol, maintaining haematopoiesis, maintaining the health of the central nervous system, and promoting the formation of connective tissue [17].

## 3. Health Benefits of Polyenoic Vegetable Oils

### 3.1. Adjunctive Lipid-Lowering Function

Inorganic acid is a functional factor in the regulation of blood lipids, which can be metabolized in the body to produce docosahexaenoic acid (DHA) and eicosapentaenoic acid (EPA). Experiments have shown that a daily dietary supply of 3–5 g of DHA and EPA is effective in reducing blood lipid levels [18]. Studies have pointed out that *α*-linoleum acid and *γ*-linoleum acid have auxiliary lipid-lowering functions for patients with hyperlipidemia and have no adverse effects on the health of the body [19].

As an essential fatty acid, linoleum acid can affect the molecular composition of plasma lipoprotein phospholipids and alter the absorption of cholesterol lipoproteins in the liver, thus having a cholesterol-lowering effect [20]. Studies have shown that linoleum acid can reduce body mass and blood lipid levels in mice, increase the activity of serum lipoprotein lipase, hepatic lipase, and total lipase, and reduce the degree of liver steatosis, which can prevent hyperlipidemia [19]. Studies have shown that diets containing oleic, linoleum, and linoleum acids reduce plasma, apolipoprotein B, and apolipoprotein A I [22], and diets high in linoleum acid reduce the elevating effect of dietary egg yolk cholesterol on serum cholesterol [23]. Therefore, polygenic vegetable oils rich in linoleum acid and linoleum acid have an adjuvant hyperlipidemia effect.

### 3.2. Antioxidant Function

Polymeric acid has a clear antioxidant function in ageing mice [24]. Vitamins can block the chain reaction of lipid peroxides in cell membranes and can effectively defend against free radical attack [25]. The trace element selenium exerts antioxidant effects through various selenium-containing proteins and selenium-containing enzymes, and selenium and VE have synergistic effects [26].

Phytosterols have potential antioxidant potential, as they inhibit oxidative degradation of oils and have a strong scavenging effect on 1,1-diphenyl-2-picrylhydrazyl (DPPH) radicals and hydroxyl radicals [27]. Therefore, polygenic vegetable oils benefit from the antioxidant effects of active substances such as polymeric acids, VE, and phytosterols. For example, peony seed oil inhibited nearly 90% of DPPH radicals and inhibited the peroxidation of unsaturated fatty acids in egg yolk and oil samples; walnut oil significantly increased the total antioxidant capacity and superoxide dismutase (SOD), catalase (CAT), and glutathione (GLUTATHIRE) in liver and brain tissues of mice.

### 3.3. Antiageing Function

The results of studies have confirmed the potential of *ω*-3 polyatomic acids to delay ageing in synergy with energy limitation or alone. The lack of EPA and DHA in Drosophila, which do not have the gene sequence encoding the Δ-5/Δ-6 desalinise enzyme, and the shortened lifespan of Drosophila after ingestion of diets supplemented with EPA and DHA were reported, but the addition of *α*-linoleum acid to the diet delayed ageing in Drosophila.

## 4. Time Series Models

In the three-layer BP network shown in Figure 1, an important feature of the network response function S function is that the derivative of the S function can be expressed by the S function itself.

(1) Initialize assign random values between (−1, +1) to each connection right {*w*_*ij*_}, {*v*_*jt*_} and threshold {*θ*_*j*_}, {*γ*_*t*_}.
(2) Randomly select a pattern pair *A*_*k*_ = (*a*_1_, *a*_2_,…, *a*_*n*_), *Y*_*k*_ = (*y*_1_, *y*_2_,…, *y*_*q*_) to provide to the network.
(3) Input learning mode “down propagation process”: input mode *A*_*k*_ = (*a*_1_, *a*_2_,…, *a*_*n*_), connection rights {*w*_*ij*_}, and threshold {*θ*_*j*_} to calculate the input of each unit in the middle layer and then {*S*_*j*_} to calculate the output of each unit in the middle layer by the S function {*b*_*j*_}:
  (1) $$\begin{array}{c} s_{j}=\overset{n}{\underset{i=1}{\sum }}w_{ij}\cdot a_{i}+\theta ,\\ j=1,2,\cdots ;p,\\ b_{j}=f\left(s_{j}\right),\\ j=1,2,\cdots ;p. \end{array}$$
(4) Compute the input {*b*_*j*_} of each unit in the output layer using the output {*v*_*jt*_} of the intermediate layer, the connection right {*γ*_*t*_}, and the threshold {*L*_*t*_} and then compute the response {*L*_*t*_} of each unit in the output layer by the S function using {*C*_*t*_}:
  (2) $$\begin{array}{c} L_{t}=\overset{p}{\underset{j=1}{\sum }}v_{jt}\cdot b_{j}-t_{t}\gamma \;t=1,2,\cdots ;q,\\ C_{t}=f\left(L_{t}\right)\;t=1,2,\cdots ;q. \end{array}$$
(5) Using the desired output pattern *Y*=(*y*_1_^*k*^, *y*_2_^*k*^, ⋯; *y*_*q*_^*k*^), the actual output of the network {*C*_*t*_}, calculate the generalized error of each cell in the output layer {*d*_*t*_^*k*^}:
  (3) $$\begin{array}{c} d_{t}^{k}=\left(y_{t}^{k}-C_{t}\right)C_{t}\left(1-C_{t}^{k}\right)\;t=1,2,\cdots ;q. \end{array}$$
(6) Calculate the generalized error {*v*_*jt*_} of each unit in the middle layer by using the connection weight {*d*_*t*_^*k*^}, the generalized error {*b*_*j*_} of the output layer, and the output {*e*_*j*_^*k*^} of each unit in the middle layer:
  (4) $$\begin{array}{c} e_{j}^{k}=\left[\sum_{t=1}^{a}d_{t}v_{jt}\right]\cdot b_{j}\left(1-b_{j}\right)\;j=1,2,\cdots ;p,\\ v_{jt}\left(N+1\right)=v_{jt}\left(N\right)+\alpha d_{t}^{k}b_{j},\\ j\neq ,2,\cdots ;p\;t\neq ,2,\cdots ;q\;\left(0<\beta <1\right)\\ \gamma \left(N+1\right)=\gamma \left(N\right)+\alpha d_{t}^{k}\;t=1,2,\cdots ;q. \end{array}$$
Using the generalized error {*e*_*j*_^*k*^} for each cell in the intermediate layer, the input correction connection weights {*w*_*ij*_} for each cell in the input layer and the threshold {*θ*_*j*_}.
  (5) $$\begin{array}{c} w_{ij}\left(N+1\right)=w_{ij}\left(N\right)+\beta e_{j}^{k}._{\alpha }\\ i=1,2,\cdots ;n,j=1,2,\cdots ;p\\ \rho \left(N+1\right)=\theta \left(N\right)+\beta e_{j}^{k}\;j=1,2,\cdots ;p. \end{array}$$
(8) Training process: randomly select the next pattern pair to be provided to the network; return to step (3), until all *m* pattern pairs are trained.

In the BP algorithm, the rules for changing the connection weights are obtained:

(6) $$\begin{array}{c} \Delta_{t}\gamma =\alpha d_{t}^{k}\;t=1,2,\cdots ;q,\\ \Delta \theta =\beta e_{j}^{k}\;j\neq ,2,\cdots ;p. \end{array}$$

The choice of *η* is very important. If *η* is chosen to be small, the learning speed of the network is not only slow but also easy to make the network fall into the local minimum; while if *η* is chosen to be too large, the network will easily oscillate and the error E will not reach the minimum. As the network learns, the learning factor *η* is changed according to the change of the learning error, and let *n* be the number of learning time; we have

(7) $$\begin{array}{c} \eta =\left(\begin{array}{c} \left(1-005\right)\eta E_{n+1}\leq E_{n}\\ \left(1+005\right)\eta E_{n+1}>1 \end{array}\right). \end{array}$$

The predict values are shown in Table 1.

The general form of the predicted value is

(8) $$\begin{array}{c} x_{t}=c_{i}x_{t-1}+c_{2}x_{t-2}+...+c_{p}x_{t-p}+\varepsilon_{t}, \end{array}$$

where {*ε*_*t*_} is the white noise and *c*_*i*_ is the constant factor.

For the same prediction problem, according to the aforementioned neural network model, the general form of the prediction value is

(9) $$\begin{array}{c} X_{t}=f_{1}\left(X\right)X_{t-1}+f_{2}\left(X\right)X_{t-2}+\cdots +f_{p}\left(X\right)X_{t-p}+\varepsilon_{t}, \end{array}$$

where *p* is the number of input nodes to the prediction network.

(10) $$\begin{array}{c} f_{i}\left(X\right)=f_{i}\left(X_{t-1},X_{t-2},\cdots ;X_{t-p},\varepsilon_{t}\right),\left(i=1,2,...,p\right), \end{array}$$

is a nonlinear function with each input variable of the prediction network as the independent variable.

The estimated value of *X*_*t*_ is

(11) $$\begin{array}{c} X_{t}=f_{1}\left(X\right)X_{t-1}+f_{2}\left(X\right)X_{t-2}+\cdots +f_{p}\left(X\right)X_{t-p}. \end{array}$$

The prediction error is

(12) $$\begin{array}{c} \sigma^{2}=\sum {\left(X_{\hat{t}}-X_{t}\right)}^{2}. \end{array}$$

The training process of neural network is not only the process of making *σ*^2^ reach the global minimum but also the establishment process of prediction model. From a statistical point of view, the final result of neural network modeling is to find the nonlinear function *f*_*i*_(*x*), and *f*_*i*_(*x*) is expressed by the connection weight threshold of each node in the network [28–30].

## 5. Experimental Analysis of ANN Prediction Modeling for the Assessment of Health Benefits of Polyenoic Vegetable Oils

After ANN network training was completed, the actual health effects of polymeric acid vegetable oils for each month of a given epidemic year were used to predict the incidence rate for each month of the next epidemic year. As shown in Figure 2, using the prediction step *K* = 12, the actual health efficacy assessment of polymeric acid vegetable oil for each month from 1992.9 to 1993.8 was used as the input of the sample, and the predicted health efficacy assessment of polymeric acid vegetable oil for each month from 1993.9 to 1994.8 was obtained.

A dynamic learning ratio ANN prediction model was used with the monthly PAO health effects assessment as the predictor, but with a different input sample than the model described above. To predict the health effects of monthly polygenic vegetable oils for the prevalent years 93.9 to 94.8, the input samples could be two segments 92.9 to 93.8 and 92.8 to 93.7, or three segments 92.9 to 93.8, 92.8 to 93.7, and 92.7 to 93.6, or four segments 92.9 to 93.8, 92.8 to 93.7, 92.7 to 93.6, and 92.6 to 93.5… After testing and screening, the best prediction results were obtained when the input sample was evaluated for the health efficacy of seven stages of lunar polymeric acid vegetable oil, with a model structure of 7-6-12 and a global error of E = 2.5 × 10^−4^, see Figure 3.

As can be seen from the figure, ANN prediction model 2 achieved satisfactory results for the assessment of the health benefits of polyenoic vegetable oils, but the model did not learn the singular values (i.e., outliers) satisfactorily.

The essential oil of peony blossom has a natural fragrance and a small molecular structure, which makes it easily absorbed. Combining peony blossom essential oil with peony seed oil can complement the advantages of peony blossom essential oil and peony seed oil, making the blend combine the advantages of both oils. Because of the high cost of peony flower essential oil and the fact that the essential oil should not be used alone and requires some dilution, the proportion of peony flower essential oil in the blend was kept below 30% in this study.

There were no inhibition circles when the ratio of peony flower essential oil to peony seed oil was 5 : 95, 10 : 90, and 1585, and there were smaller inhibition circles when the ratio was 20 : 80, 25 : 75, and 30 : 70. From Table 2, it can be seen that the diameter of the inhibition circle of the six different mix ratios of the oil mix is as follows: mix ratio of 30 : 70> mix ratio of 25 : 75> mix ratio of 20 : 80> mix ratio of 15 : 85, 10 : 90, and 5 : 95, where the mix ratio of 15 : 850 : 90 and 5 : 95 inhibition circle diameter of the oil mix is not significantly different (*P* < 0.05).

UV rays are very penetrating and can cause damage to the skin over a long period of time. Depending on the degree of damage to the skin, UV rays can be divided into 3 wavelengths: the short wavelength of 200–280 nm, the medium wavelength of 280–320 nm, and the long wavelength of 320–400 nm.

As can be seen from Figure 4, the absorption capacity of different proportions of peony flower essential oil and peony seed oil blends for different wavelengths of UV light all showing a trend of rising and then falling. When the wavelength was 280–300 mil, the absorption value of UV light did not change much when the oil was mixed with different ratios. However, when the wavelength was 310–400 mm, the peak value of the UV absorption of the oil mixture shifted to the right as the proportion of peony flower essential oil increased. When the wavelength was 280–400 nm, the absorption values of the six different oil blends were as follows: 30 : 70 oil blends >25 : 75 oil blends >20 : 80 oil blends >15 : 85 oil blends >1090 oil blends >5 : 95 oil blends.

As can be seen from Table 3, the weights of each evaluation factor of peony flower essential oil-seed oil blend were light transmission and color (0.0966) aroma (0.0767), dispersibility (0.1080), absorption (0.1932), smoothness (0.0739), residual sensation (0.1364), UV resistance (0.173), and antibacterial effect (0.1420). That is, *A* = {0.0966, 0.0767, 0.1080, 0.1932, 0.0739, 0.1364, 0.1733, 0.1420}. The highest weights were given to absorbency, UV resistance, and antibacterial effect among the eight factors, indicating that the tested population placed more importance on the absorbency, UV resistance, and antibacterial effect of the base oils for cosmetics.

## 6. Conclusions

Most of the current research on polymeric vegetable oils at home and abroad is focused on the screening of oil species, optimization of extraction methods, analysis of fatty acid composition, research on health effects, etc. Some vegetable oils, such as peony seed oil, have been used in the preparation of health food or skin care and beauty products. Considering the low production of these oils, their high price and the fact that they are rich in essential fatty acids such as linoleum acid and linoleum acid and are susceptible to oxidation, it is recommended that more efforts be made in the research and development of technologies, such as efficient extraction, antioxidation, separation and purification, oil modification, ultrafine treatment, and comprehensive utilization, and that the development of new varieties, testing of active ingredients. The research and development of new varieties and testing of active ingredients and functional properties will be strengthened to broaden the scope of new functions and applications and increase the added value.

China is rich in polygenic vegetable oil resources, and compared with ordinary vegetable oil, its nutritional value and health effects are more prominent. It is a kind of natural functional vegetable oil, which can be widely used in nutritional and healthy edible oil, health food, skin care, beauty cosmetics, etc., and will have a broad development and utilization prospect.

## Figures and Tables

**Figure 1:** Three-layer BP network structure.

**Figure 2:** Prediction curve for the assessment of health benefits of HFRS monthly polyenoic vegetable oils in the ANN model 1 prevalence year (*K* = 12).

**Figure 3:** Predicted curves for the assessment of health benefits of HFRS monthly polyenoic vegetable oils in the ANN model 4 prevalence years (*K* = 12).

**Figure 4:** UV resistance of oil blends of different proportions.

**Table 1:** Segmentation method for training data.

*N* inputs	*M* outputs
*X*_1_, *X*_2_, ⋯, *X*_*N*_	*X*_*N*_+1, *X*_*N*+2_, ⋯; *X*_*N*+*M*_
*X*_2_, *X*_3_, ⋯, *X*_*N*+1_	*X*_*N*+2_+1, *X*_*N*+3_, ⋯; *X*_*N*+*M*+1_
*X*_3_, *X*_4_, ⋯, *X*_*N*_+2	*X*_*N*+3_, *X*_*N*+4_, ⋯, *X*_*N*+*M*+2_
*X*_*K*_, *X*_*K*_+1, ⋯, *X*_*N*_+*K* − 1	*X*_*N*+*K*_, *X*_*N*+*K*+1_, ⋯, *X*_*N*+*M*+*N*−1_

**Table 2:** Different proportions of mixed oils.

Strain	*Staphylococcus aureus*					
Mixture ratio	5 : 95	10 : 90	15 : 85	20 : 80	25 : 75	30 : 70
Bacteriostatic ring diameter (mm)	6.00 ± 0.00^*d*^	6.00 ± 0.00^*d*^	6.00 ± 0.00^*d*^	7.12 ± 0.02^*c*^	7.22 ± 0.02^*b*^	7.37 ± 0.04^*a*^

**Table 3:** Summary of weights.

Evaluation factors	Comparison results									
	Light transmittance and color	Aroma	Dispersibility	Absorptivity	Smoothness	Residual sense	UV resistance	Bacteriostatic effect	Total score	Weight
Light transmittance and color	10	4	6	0	6	2	2	4	34	0.108
Aroma	6	9	1	0	6	2	1	2	27	0.0767
Dispersibility	5	8	10	1	8	3	1	2	38	0.108
Absorptivity	10	10	9	10	10	8	5	6	68	0.1923
Smoothness	4	4	4	0	10	2	1	1	26	0.0739
Residual sense	7	8	5	2	9	10	2	5	48	0.1364
UV resistance	8	8	8	5	9	7	9	7	61	0.1733
Bacteriostatic effect	6	8	5	5	8	6	2	10	50	0.142

## Data Availability

The data underlying the results presented in the study are available within the article.
